# *Egr1* mediates retinal vascular dysfunction in diabetes mellitus via promoting p53 transcription

**DOI:** 10.1111/jcmm.14225

**Published:** 2019-03-19

**Authors:** Haocheng Ao, Bingqian Liu, Haichun Li, Lin Lu

**Affiliations:** ^1^ State Key Laboratory of Ophthalmology Zhongshan Ophthalmic Center, Sun Yat‐sen University Guangzhou China

**Keywords:** diabetic retinopathy, Egr1, p53

## Abstract

**Objectives:**

This study focused on investigating the expression and underlying molecular mechanism of early growth response 1 (*Egr1*) in diabetic retinopathy.

**Methods:**

A microarray assay was applied to examine differentially expressed genes in the retina tissues of normal rats, as well as in those of streptozotocin‐induced diabetic rats. Human retinal vascular endothelial cells (HRVECs) transfected with sh‐NC, sh‐*Egr1* or sh‐*Egr1*+ pVax1‐p53 were cultured under high‐glucose conditions and then used to explore the role of *Egr1 *in vitro. The effect of *Egr1* on retinal vascular dysfunction caused by diabetes was examined by sh‐*Egr1* administration in vivo

**Results:**

Early growth response 1 was found to be up‐regulated in the retinas of diabetic rats compared to those of normal rats. Down‐regulation of *Egr1* in HRVECs under high‐glucose conditions inhibited the apoptosis, migration and tube formation in vitro. Moreover, sh‐*Egr1* partially reduced the injurious effects of hyperglycaemia on retinal vascular function by decreasing apoptotic cells and microvascular formation in vivo. The reduction of *Egr1* evidently down‐regulated the p53 expression. Overexpression of p53 rescued the inhibition of sh‐*Egr1* in HRVECs under high‐glucose concentration on apoptosis, migration and tube formation in vitro.

**Conclusion:**

Down‐regulation of *Egr1* partially reduced the injurious effects of hyperglycaemia on retinal vascular function via inhibiting p53 expression.

## 1 INTRODUCTION

Retinopathy is one of the most common and severe diabetic complications. Diabetic retinopathy (DR) remains one of the major causes of vision impairment and even blindness in working‐age people worldwide.^1^ Diabetic retinopathy, which is a neurodegenerative illness, is a gradual deterioration that leads to cellular lesions of a wide range of retinal cells.^2^ One of the early functional changes of DR is pericyte loss. Subsequently, vision‐threatening conditions in DR are caused by macular oedema and neovascularization.^3^ Diabetic retinopathy aggravates diabetic patient conditions in spite of the recent improvements in the treatment of DR via photocoagulation and glycaemic control.^3^ Accordingly, further studies that focus on the mechanism of DR progression are needed, which may help researchers understanding the molecular mechanisms that drive the vascular complications/dysfuction of DR and provide effective strategies for the treatment of DR.

Early growth response 1 (*Egr1*) has been defined as a zinc finger transcription factor of 59 kDa, rarely existing in the regulation of DNA‐binding transcription.^4^ As an important transcription factor, *Egr1* has been revealed to play significant role in diverse pathways, such as activating growth and differentiation or the transcription of target genes.^5^ Contrary to the activating growth function, overexpression of *Egr1* inhibited the cell proliferation and promoted apoptosis, and knocking out *Egr1* promoted cell proliferation.^6^ All of these indicate that the effects of *Egr1* are complicated and may depend on the type of disease.

Numerous studies have shown that the expression of *Egr1* is dramatically triggered by hyperglycaemia in diabetes mellitus. Aljada et  al found that high‐glucose intake can increase the expression of *Egr1* and tissue factor (TF), which regulates the processes that are potentially relevant to atherosclerotic plaque rupture and thrombosis.^7^ High expression of *Egr1* resulting from insulin and glucose in vascular cells may be one of the initial key events that plays a critical role in the development of the vascular complications of diabetes.^8^ Furthermore, the mRNA level of EGR1 was significantly increased in STZ‐induced diabetic mice after 6 weeks of induction.^9^ Most importantly, Karthikkeyan first reported that hyperglycaemia enhanced the *Egr1* expression in human retinal endothelial cells, mediating vascular dysfunction by regulating the expression of TF and ICAM‐1.^10^ However, the biological function and regulatory mechanism of *Egr1*, particularly in DR, remains far from fully understood.

A well‐known tumour suppressor gene, p53, is paramount in the regulation of cell differentiation and cell cycle and the mediation of cell apoptosis.^11^ It was reported by Lim et  al that p53 exhibited significant up‐regulation in the conjunctiva of diabetic patients compared to that of non‐diabetic patients.^11^ Kim et  al reported that hyperglycaemia decreased Glucagon‐like peptide‐1 receptor (GLP‐1R) expression in retinal pigment epithelial (RPE) cells and decreased the generation of intracellular reactive oxygen species, which increased ER stress‐mediated p53 expression, and subsequently caused apoptosis by increasing Bax promoter activity.^12^ In accordance with the general overview of recent studies, p53 and multiple other tumour suppressors, such as transforming growth factor β1‐(TGFβ1), phosphatase and tensin homolog and fibronectin, can be directly regulated by *Egr1*.^4^ Interestingly, p53 was found to promote the expression of *Egr1* and lead to apoptosis of A549 cells, suggesting a complex regulation of *Egr1* and p53 in vitro.^13^ Therefore, it is of great significance to explore the correlation between the p53 pathway and *Egr1*, particularly in DR.

In this study, we investigated the expression and regulatory mechanism of *Egr1* in diabetic retinopathy in vitro and in vivo, and found that *Egr1* was augmented after the induction of hyperglycaemia and that *Egr1* regulated retinal endothelial cell apoptosis, migration and vascularization by promoting p53 transcription.

## 2 MATERIALS AND METHODS

### 2.1 Streptozotocin‐induced diabetic rats

Animals were housed in a specific pathogen‐free facility and maintained according to the guidelines of the Care and Use of Laboratory Animals (published by the National Institutes of Health, NIH publication no. 86‐23, revised 1996). All rats were maintained by the Animal Laboratory of the State Key Laboratory of Ophthalmology, Zhongshan Ophthalmic Center, Sun Yat‐sen University (Guangzhou, China). Animal care and experiments complied with the ARRIVE guidelines and were in accordance with the UK Animals (Scientific Procedures) Act, 1986 and associated guidelines, EU Directive 2010/63/EU for animal experiments and approved by the Institutional Animal Care and Use Committee of State Key Laboratory of Ophthalmology, Zhongshan Ophthalmic Center, Sun Yat‐sen University.

Male Sprague‐Dawley (SD) rats (160‐180 g) were procured from Southern Medical University (Guangzhou, China). Rats were fasted for 6 hours prior to streptozotocin (STZ, Sigma, St. Louis, MO) injection. They received an intraperitoneal injection (IP) of STZ (50 mg/kg) or vehicle (citrate buffer control) for five consecutive days. The fasting blood glucose was determined using a glucometre (Precision PC; Medic, Cambridge, UK) at 7 days after the last STZ injection. A plasma glucose level in SD rats above 15 mmol/L was considered hyperglycaemic (diabetic). At the time of retinal harvest, rats were given a lethal dose (100 mg/kg) of pentobarbital (Ovation Pharmaceuticals Inc, Deerfield, IL) by IP. Retinas were excised, quickly frozen in liquid nitrogen and stored at −80°C prior to the subsequent experiments, following a protocol.

### 2.2 Illumina microarray analysis of mRNA expression

Microarray analysis was performed using Illumina Ref8 microarrays. For the STZ experiment, n = 8 control and n = 6 STZ‐treated animals were analysed. Samples were labelled according to the Illumina TotalPrep RNA Amplification kit (Illumina, San Diego, CA) standard procedures. R language was used to analyse the differentially expressed genes, and Kyoto Encyclopedia of Genes and Genomes (KEGG) enrichment analysis was applied to investigate the dysregulated pathways. *P* < 0.05 and |log_2 _(FC)| > 1 were used as the threshold to screen up‐regulated and down‐regulated mRNA.

### 2.3 RNA isolation and quantitative reverse transcription‐PCR

Total RNAs in cells and retinas were extracted using TRIzol reagent. NanoDrop ND1000 was used for qualitative and quantitative analysis for total RNAs. A quantity of 1 µg total RNA was transcribed into cDNA using the PrimeScript RT Master Mix. Then, the SYBR Premix Ex Taq II kit was used for quantitative PCR. All the transcriptional and PCR kits were obtained from Takara (Dalian, China). The relative quantification values of the mRNAs were normalized to the control using the 2^−ΔΔct^ method, and the internal control for the mRNA was GADPH. The quantitative reverse transcription‐PCR (qRT‐PCR) primer sequences were as follows: *Egr1* forward primer: 5′‐CTGACCGCAGAGTCTTTTCCTG‐3′, and reverse primer: 5′‐TGGGTGCCGCTGAGTAAATG‐3′; p53 forward primer: 5′‐TGTCATGGCGACTGTCCAGC‐3′, and reverse primer: 5′‐GCTCGACGCTAGGATCTGAC‐3′; glyceraldehyde‐3‐phosphate‐dehydrogenase (GAPDH) forward primer: 5′‐TGCACCACCAACTGCTTAGC‐3′, and reverse primer: 5′‐GGCATGGACTGTGGTCATGAG‐3′.

### 2.4 Western blots

Radio‐immunoprecipitation assay buffer (Beyotime, Shanghai, China) was applied to lyse the cells or tissues to obtain total protein. Then, the protein was quantified with the BCA Protein Assay Kit (Beyotime) following the conditions suggested by the manufacturer. A quantity of 40 μg of total protein was used for SDS‐PAGE followed by electrophoretic transfer onto polyvinylidene difluoride (PVDF) membranes. After blocking, the membranes were incubated with an anti‐GAPDH antibody (ab181603, 1:1000; Abcam, Cambridge, UK), rabbit polyclonal anti‐Fas antibody (ab82419, 1:1000; Abcam), rabbit polyclonal anti‐p53 antibody (ab61241, 1:1000; Abcam) or rabbit polyclonal Anti‐*Egr1* antibody (ab208780, 1:1000; Abcam) in TBST containing 5% non‐fat milk overnight at 4°C. After washing three times with TBST, the membranes were incubated with a goat polyclonal to rabbit IgG H&L (HRP) pre‐adsorbed (ab7090; Abcam, Cambridge, MA) at a dilution of 1:2000 in phosphate‐buffered saline with 0.1% Tween 20 (PBST) for 1 hour at room temperature (RT). The membranes were subsequently washed three times with PBST, and the electrochemiluminescence plus system (Beyotime) was used to visualize the protein bands. The density of the immunoblot was analysed using the Lab Works 4.5 software (Ultra‐Violet Products, Cambridge, UK).

### 2.5 Construction of Egr1 and p53 overexpression plasmids

To construct a wild‐type *Egr1* expression vector, *Egr1* gene cDNA was amplified by PCR using PBMC cDNA as template. The following primers were synthesized according to the sequence of the* Egr1* gene (NM_001964) obtained from GeneBank with *Eco*RI and *Xho*I restriction enzyme sites introduced and were used at the indicated annealing temperatures: *Egr1* sense: 5′‐GCGAATTCATGGCCGCGGCCAAGGCCGA‐3′ (271‐290), and antisense: 5′‐GGCTCG AGTTAGCAAATTTCAATTGT‐3′ (1885‐1902) (restriction sites underlined) at 60°C for 30 cycles; the predicted band was 1632 bp. The PCR products were then inserted into the *Eco*RI and *Xho*I sites of the pVax1 vector and named pVax1‐*Egr1*. The pVax1‐p53 vector was constructed following a similar procedure. All recombinant plasmids described above were verified by DNA sequencing (BioAsia Bioengineering Inc, Shanghai, China).

### 2.6 Cloning and production of *Egr1* shRNA‐containing adeno‐associated virus

Oligonucleotides encoding shRNAs directed against *Egr1* were cloned to the BglII/HindIII‐cut backbone fragment of pSUPER‐hSyn‐EGFP‐CytB‐AS to obtain pSUPER‐hSyn‐EGFP‐H1‐*Egr1* shRNA. The sequences of the shRNA primers were as follows: sh‐*Egr1*‐sense: GATCCATGCGTAACTTCAGTCGTAAGAGAACTTTACGACTGAAGTTACGCATTTTTTTCTCGAGA‐3′; sh‐*Egr1*‐antisense: 5′‐AGCTTCTCGAGAAAAAAATGCGTAACTTCAGTCGTAAAGTTCTCTTACGACTGAAGTTACGCATG‐3′. The insert containing the H1‐promoter and the shRNA were cut out from these vectors. Different serotypes of adeno‐associated virus (AAV) differ in their tropism, or the types of cells they infect. As the AAV serotype DJ is the leading candidate vector for retina transduction, we chose AAV‐DJ (type 2/type 8/type 9 chimera) and cloned the shRNA or scrambled sequences into this vector (pAAV‐U6‐GFP‐shRNA). For AAV production, vectors were cotransfected with the pAAV‐RC1 and pHelper vectors in the 293T packaging cell line (Cell Biolabs). Forty‐eight hours after transfection, cells were harvested and AAVs were purified by ultracentrifugation.

### 2.7 Cell culture and transfection

Human retinal vascular endothelial cells (ScienCell Research Laboratories, Carlsbad, CA) were cultured in high‐glucose (HG, with 4500.0 mg/L dextrose) or basic (with 1000.0 mg/L dextrose) DMEM medium (Invitrogen, Carlsbad, CA) containing 10% (v/v) foetal bovine serum (FBS; Gibco, Grand Island, NY). Two‐hundred and ninety three T cells were obtained from ATCC (Manassas, VA) and cultured in basic DMEM medium supplemented with 10% FBS under the condition of 37°C and 5% CO_2_. These cells were transfected with sh‐NC, sh‐*Egr1*, pVax1‐*Egr1*, or pVax1‐p53 using LipofectamineTM 2000 (Life Technologies, Carlsbad, CA) on the basis of the manufacturer's protocol.

### 2.8 Dual Luciferase reporter assay

The p53‐Luc reporter plasmids were purchased from Stratagene (La Jolla, CA). Two‐hundred and ninety three T cells were seeded into 96‐well plates (5 × 103 cells/well) at 24 hours before transfection. The cells were cotransfected with a mixture of the firefly luciferase reporter vector, pRL‐TK (Renilla Luciferase Control Reporter Vectors) (Promega, Madison, WI), and either pVax1‐*Egr1* or sh‐*Egr1*. At 48 hours post‐transfection, the luciferase activity was detected using a dual luciferase reporter assay system (Promega).

### 2.9 Apoptosis assay

The extent of apoptosis was assessed by annexin V‐FITC and propidium iodide (PI) double staining. Briefly, cells were harvested, washed twice with PBS and re‐suspended at 1 × 10^6^ cells/mL in 100 μL binding buffer. Cells were incubated with annexin V‐FITC and PI for 15 minutes at RT in the dark and mixed with 400 μL binding buffer. Then, the cells were analysed using FACScan (BD Biosciences, San Jose, CA), and apoptotic rates were measured using FlowJo 6.0 software.

### 2.10 Wound‐healing assay

Cell lateral migration was analysed in vitro using a wound‐healing assay. In brief, HRVECs under high‐glucose conditions were transfected with sh‐NC, sh‐*Egr1*, sh‐*Egr1*+pVax1 or sh‐*Egr1*+pVax1‐p53. After 24 hours of transfection, those cells were cultured in 12‐well plates to near confluence and starved in HG DMEM medium with 0.2% FBS for 12 hours. A scratch was created in each well with a 200‐µL tip. After rinsing, cell migration in the scratched area was monitored by phase‐contrast microscopy at 24 hours after transfection. Considering the effects of glucose concentration on cellular function, HRVECs under basic‐glucose conditions were also used as a control. The percentage of migrated cells within the original scratch was quantified using ImageJ.

### 2.11 Cell migration assay

The migration assays were conducted using transwell chambers according to the manufacturer's protocol (BD Science, Bedford, MA). At 24 hours after transfection with sh‐NC, sh‐*Egr1*, sh‐*Egr1*+ pVax1 or sh‐*Egr1*+ pVax1‐P53, HRVECs were trypsinized and suspended in 100 μL HG DMEM (5 × 10^4^ cells) containing 1% FBS, then were added to the upper chambers. High‐glucose DMEM supplemented with 10% FBS was added to the bottom wells of the chambers. After 6 hours of incubation, cells on the upper side of the membrane were then removed, while the cells that had migrated through the membrane to the underside were fixed and stained with 0.1% crystal violet. Cell numbers were counted in five random fields at 200× magnification using light microscopy. The data were expressed as the mean value of cells in five fields based on three independent experiments. Migration rate was expressed as the fold change (FC) of the number of migrated cells through a transwell plate.

### 2.12 Tube formation assay

The formation of capillary‐like structures was detected in a 24‐well plate using growth factor‐reduced Matrigel (BD Biosciences). After transfection with sh‐NC, sh‐*Egr1*, sh‐*Egr1*+ pVax1 or sh‐*Egr1*+ pVax1‐P53, HRVECs (1 × 10^5^ cells/well) were plated onto Matrigel (300 μL/well). After 24 hours of cell culture, these cells were observed using a bright‐field microscope. The tube length was quantified using ImageJ software.

### 2.13 Intravitreal injection

At the beginning of diabetes induction, diabetes rats were anaesthetized by IP of ketamine (80 mg/kg) and xylazine (4 mg/kg). Approximately 1.5 μL (1 × 10^12^ vg/mL) of AAV containing sh‐*Egr1* and sh‐NC was delivered into the vitreous body using a 33‐gauge needle. To maximize virus delivery, rats received an intravitreal injection every 10 days. The rats were sacrificed, and the retinas were harvested at two months after injection.

### 2.14 Terminal dUTP nick‐end labelling assay for detection of apoptotic nuclei

For the retinal cell apoptosis analysis, the terminal dUTP nick‐end labelling (TUNEL) assay was carried out with the tetramethylrhodamine (TMR) red cell death detection kit (Roche, Mannheim, Germany) according to the manufacturer's instructions. In brief, eye cryosections were fixed with 4% paraformaldehyde (PFA) at RT for 10 minutes and then immersed in ethanol/acetic acid (2:1) for 5 minutes at −20°C. Subsequently, sections were washed twice with cold PBS (pH 7.4) for 5 minutes. The washed sections were sequentially catalysed with digoxigenin‐dNTP and then stained with TUNEL In Situ Cell Death Detection kit. Processed slides were mounted with Vectashield mounting medium containing DAPI (Vectashield; Vector, Burlingame, CA) and viewed using a fluorescence microscope (Axioplan2; Carl Zeiss Meditec, Inc., Dublin, CA).

### 2.15 Statistical analysis

All quantitative values were presented as the mean ± SD. The differences among the groups were analysed by one‐way ANOVA using GraphPad Prism v6.0 (GraphPad Software, Inc., San Diego, CA). *P* < 0.05 was considered statistically significant.

## 3 RESULTS

### 3.1 *Egr1* was highly expressed in the retinas of rats with DR

In an effort to screen differentially expressed genes in the retinas of STZ‐induced diabetic rats and those of normal rats, we used a *t* test (*P < *0.05) combined with FC >2 to screen up‐regulated and down‐regulated mRNAs respectively. As shown in Figure 1A, *Egr1* was significantly up‐regulated in STZ‐induced diabetic rats’ retinal tissues. To further confirm the expression of *Egr1* in diabetes, STZ was used for the induction of diabetes in the rats. After STZ‐induction, the mRNA levels of *Egr1* were significantly increased in the retinas of STZ‐induced diabetic rats compared to those of the normal rats (Figure 1B). As hyperglycaemia in diabetics contributes to DR, we wondered whether exposing HRVECs to high glucose (25 mmol/L) would alter *Egr1* expression. The results showed that *Egr1* was evidently up‐regulated in HRVECs under high‐glucose conditions compared to basic‐glucose conditions at the mRNA (Figure 1C) and protein levels (Figure 1D,E).

**Figure 1:** Early growth response 1 (*Egr1*) is up‐regulated in diabetic retinopathy tissues and human retinal vascular endothelial cells (HRVECs) under high‐glucose (HG) conditions. A, Heat map of differentially expressed mRNAs in the retinas of normal and streptozotocin (STZ)‐induced diabetic rats. B, The diagram shows expression of *Egr1* in retinal tissues of normal and STZ‐induced diabetic rats measured by qRT‐PCR (n = 20; *P < 0.05). C, The mRNA expression of *Egr1* in HRVECs under basic and HG conditions for 2 wk (*P < 0.05 compared with Basic group). D, Protein expression of *Egr1* in HRVECs cultured in HG conditions measured by Western blot. E, Quantification analysis of *Egr1* protein expression according to Figure 1D (**P < 0.01 compared with Basic group).

### 3.2 *Egr1 *regulated endothelial cell function under high‐glucose conditions in vitro

We next investigated the role of *Egr1* in retinal endothelial cells under high‐glucose conditions. Following HRVEC transfection with *Egr1* shRNA or sh‐NC for 48 hours, the expression of *Egr1* in the sh‐*Egr1* group was dramatically lower than that of sh‐NC group (Figure 2A). In addition, the apoptosis of HRVECs determined by annexin V/PI dual‐staining assays showed that sh‐*Egr1* transfection significantly decreased HRVECs apoptosis (Figure 2B). Wound‐healing and transwell assays revealed that down‐regulation of *Egr1* by sh‐*Egr1* significantly inhibited the horizontal and vertical migration ability of HRVECs under high‐glucose conditions (Figure 2C,D). Additionally, transfection with sh‐*Egr1* evidently inhibited tube formation in high‐glucose conditions, as reflected by decreased tube length, while the tube length of the scrambled group was barely affected (Figure 2E).

**Figure 2:** Early growth response 1 (*Egr1*) regulates endothelial cell function under high‐glucose (HG) conditions in vitro. A, Human retinal vascular endothelial cells (HRVECs) under HG conditions were transfected with sh‐NC and sh‐*Egr1*. Quantitative reverse transcription‐PCR was conducted to detect *Egr1* mRNA expression (**P < 0.01). B, Flow cytometric analysis of apoptotic HRVECs cells following transfection for 48 h was conducted and the total rate of apoptosis was calculated. (**P < 0.01). C, Wound‐healing assay and quantification analysis were conducted to detect the lateral migration of HRVECs (*P < 0.05 vs Basic group; ^#^ *P* < 0.05 vs HG group). Scale bar: 100 μm. D, Transwell and quantification analysis were conducted to detect the vertical migration of HRVEC (*P < 0.05 vs Basic group; ^#^ *P* < 0.05 vs HG group). Scale bar: 50 μm. E, HRVECs were seeded on the Matrigel matrix. The formation of tube‐like structures was observed 24 h after cell seeding. Average length of tube formation for each field was statistically analysed (*P < 0.05 vs Basic group; ^#^ *P* < 0.05 vs HG group). Scale bar: 100 μm.

### 3.3 *Egr1* regulated diabetes mellitus‐induced retinal vascular dysfunction in vivo

We further investigated the role of *Egr1* in retinal vascular dysfunction in vivo. Adeno‐associated viral shRNAs targeting *Egr1* were intravitreally injected into STZ‐induced diabetic rats. Quantitative reverse transcription‐PCR revealed that sh‐*Egr1* treatment significantly blocked mRNA expression of retinal *Egr1* (Figure 3A) and *p53* mRNA (Figure 3B), and correlated with the down‐regulation of their protein levels (Figure 3C). Furthermore, the number of diabetes‐induced TUNEL (+) cells was dramatically reduced in sh‐*Egr1*‐treated rats compared with diabetic rats that received sh‐NC (Figure 3D), while most of those apoptotic cells were mainly localized in the inner nuclear layer (INL) and outer nuclear layer (ONL).

**Figure 3:** Early growth response 1 (*Egr1*) regulates diabetes mellitus‐induced retinal vascular dysfunction in vivo. (A,B) streptozotocin (STZ)‐induced diabetic SD rats received intravitreous injections of sh‐NC or sh‐*Egr1* every day for 10 d. Two months after injection, quantitative reverse transcription‐PCRs were conducted to determine *Egr1* and p53 mRNA expression (^*^ *P* < 0.05, ^**^ *P < *0.01). C, The protein levels of Egr1 and p53 in sh‐NC and sh‐*Egr1 *STZ diabetic rats. D, Cryopreserved eye sections were made from the 2‐month‐old treated and untreated diabetic rats (STZ). Cell apoptosis was detected by terminal dUTP nick‐end labelling (TUNEL) staining. Quantification of the TUNEL (+) cells were shown as the mean ± SD. Scale bar: 100 μm. ^**^ *P* < 0.01 vs sh‐NC group.

### 3.4 p53 signalling pathway was activated in DR

KEGG pathway enrichment analysis indicated the remarkable enrichments of differentially expressed genes in 14 items and demonstrated that p53 signalling pathway was activated in STZ‐induced DR (Figure 4A). Moreover, Gseaplot revealed that the running enrichment score of the p53 signalling pathway in STZ‐induced DR tissues was greater than 0, indicating that p53 signalling pathway was activated (Figure 4B). As protein‐protein interactions are important for organizing all protein coding genes in a genome, we applied String and Smartdraw to explore the pathway interactions between the genes. Our data showed that there was a direct association between *Egr1* and p53 (Figure 4C). To further clarify the effects of high glucose on p53 expression in HRVECs, incubation of HRVECs with high glucose (25 mmol/L) for 2 weeks exhibited up‐regulation of p53 mRNA levels (Figure 4D). The p53 protein expression levels examined by Western blotting revealed that p53 protein was significantly up‐regulated in HRVECs under high‐glucose conditions compared with basic‐glucose conditions (Figure 4E).

**Figure 4:** p53 signal pathway is up‐regulated in diabetic retinopathy. A, The diagram showed the name of the KEGG pathway that was significantly up‐regulated in the control and streptozotocin (STZ) groups, in which the KEGG p53 signal pathway was significantly up‐regulated. B, Gseaplot revealed that the running enrichment score of the p53 signalling pathway in the STZ groups was more than 0, indicating that the p53 signalling pathway was activated. C, Online analysis of the relationship between early growth response 1 and related proteins of the p53 signalling pathway by STRING (version 10.0). D, The mRNA expression of p53 in human retinal vascular endothelial cells (HRVECs) under high‐glucose (HG) induction for 2 wk (**P < 0.01). E, Protein expression of p53 in HRVECs cultured in basic and HG conditions for 2 wk was evaluated by Western blot.

### 3.5 *Egr1* promoted transcription and expression of p53

To directly investigate whether *Egr1* regulates p53 expression, a dual‐luciferase reporter assay was carried out. We found that *Egr1* was capable of increasing the luciferase activity driven by pVax1‐*Egr1* markedly (Figure 5A), while sh‐*Egr1* obviously decreased the luciferase activity in 293T cells (Figure 5B). HRVECs under high‐glucose conditions transfected with sh‐*Egr1* were found to down‐regulate p53 and its target gene Fas at the mRNA level (Figure 5C,E). Moreover, Western blot results indicated that the protein levels of p53 and Fas were significantly down‐regulated under high‐glucose conditions in the HRVEC group that was transfected with sh‐*Egr1* compared with the group transfected with sh‐NC and the control group (Figure 5D and 5F). Those results indicated that *Egr1* was a transcriptional regulatory factor of p53 and that it promoted p53 expression.

**Figure 5:** Expression of p53 is promoted by Early growth response 1 (*Egr1*). A, 293T cells were cotransfected with the indicated p53 promoter‐luc plasmids and plasmids expressing *Egr1* for 48 h, and luciferase activity was measured (***P < 0.001). The DNA binding domain of Egr1 on p53 gene were shown in the upper part. B, 293T cells were cotransfected with the indicated p53 promoter‐luc plasmids and sh‐NC or sh‐*Egr1* for 48 h, and luciferase activity was measured (**P < 0.01). C, Relative mRNA expression of p53 after transfection was detected by quantitative reverse transcription‐PCR (qRT‐PCR) (***P < 0.001 vs pVax1 group; ^#^ *P < *0.05 vs sh‐NC group). D, Protein expression of p53 transfected with pVax1‐p53 or sh‐*Egr1* in human retinal vascular endothelial cells (HRVECs) under HG were measured by Western blot. E, Relative mRNA expression of Fas after transfection was detected by qRT‐PCR (***P < 0.001 vs pVax1 group; ^#^ *P < *0.05 vs sh‐NC group). F, Protein expression of Fas transfected with pVax1‐p53 or sh‐*Egr1* in HRVECs under HG was measured by Western blot.

### 3.6 *Egr1* regulated retinal endothelial cell function via the induction of the expression of p53 in HRVECs

To confirm the role of *Egr1* on mediating the activation of p53 in high‐glucose conditions, we transfected HRVECs with sh‐*Egr1*, which reduced *Egr1* protein expression (Figure 6A). The ability of sh‐*Egr1* to suppress the activation of p53 was significantly suppressed in pVaxl‐p53‐transfected cells (Figure 6A). The statistical results of the annexin V/PI staining assays demonstrated that sh‐*Egr1* transfection notably hampered HRVECs apoptosis, while p53 overexpression obviously facilitated cell apoptosis in the sh‐*Egr1*+pVax1‐p53 group compared with the sh‐*Egr1* group (Figure 6B). Based on the transfections with sh‐*Egr1*, we treated the HRVECs with pVax1‐p53, which increased cell migration compared with sh‐*Egr1* transfection alone (Figure 6C,D). pVax1‐p53 obviously increased tube length, although the HRVECs had been transfected with sh‐*Egr1* in high‐glucose conditions (Figure 6E). These results suggested that repressing *Egr*1 expression relieved the effects of high glucose on retinal endothelial cell function via the inhibition of p53 transcription.

**Figure 6:** Early growth response 1 (*Egr1*) regulates endothelial cell function through promoting transcription of p53 in vitro. A, Western blot of p53 proteins in human retinal vascular endothelial cells (HRVECs) under high‐glucose (HG) conditions with sh‐NC, sh‐*Egr1*, sh‐*Egr1*+ pVax1 or sh‐*Egr1*+ pVax1‐P53. B, The apoptosis of HRVECs under HG condition was monitored by annexin V/PI flow cytometry under different transfection conditions (^*^ *P* < 0.05 vs sh‐NC group; ^#^ *P* < 0.05 vs sh‐*Egr*1 group). C, A wound‐healing assay was used to measure lateral migration of HRVECs under HG conditions under different transfection conditions (**P < 0.01 vs sh‐NC group; ^#^ *P* < 0.05 vs sh‐*Egr1* group). Scale bar: 100 μm. D, A transwell assay was performed to measure the vertical migration of HRVECs under HG conditions under different transfection conditions (**P < 0.01 vs sh‐NC group; ^##^ *P* < 0.01 vs sh‐*Egr1* group). Scale bar: 50 μm. E, HRVECs were seeded on a Matrigel matrix. The formation of tube‐like structures was observed 24 h after cell seeding. Average length of tube formation in each field was statistically analysed (*P < 0.05 vs sh‐NC group; ^#^ *P* < 0.05 vs sh‐*Egr1* group). Scale bar: 100 μm.

## 4 DISCUSSION

In the present study, we investigated the role of *Egr1* in DR. Up‐regulation of *Egr1* was observed in the retinas of diabetic rats. We demonstrated that *Egr1* could regulate vascular endothelial cell function in vitro and diabetes mellitus‐induced retinal vascular dysfunction in vivo through enhancing the transcription and expression of p53.

Up‐regulation of *Egr1* in diabetes‐related diseases has been noted in numerous studies. Early growth response protein 1 has been shown to participate in diabetic nephropathy through enhancing ECM production and MC proliferation and by interacting with TGF‐β1.^14^ Moreover, prolonged expression of *Egr1* contributes to prothrombotic and pro‐inflammatory responses in diabetic atherosclerosis.^15^ Additionally, hyperglycaemia‐induced *Egr1* expression in the retinal endothelium is involved in diabetes‐mediated retina vascular aberration via the up‐regulation of downstream genes.^10^ By performing microarray analysis in STZ‐induced retina specimens, we observed that *Egr1* was up‐regulated. Consistent with the results of microarray analysis, the mRNA and protein levels were increased in HG‐induced HRVECs in vitro. Early growth response protein 1 expression under hyperglycaemic conditions tends to become up‐regulated such that *Egr1* may be involved in the pathological changes of DR.

Diabetic retinopathy includes non‐proliferative (NPDR) and proliferative (PDR) forms of the disease. Prolonged hyperglycaemia is largely responsible for the development of NPDR.^1^ Apoptotic death of vascular cells mediated by hyperglycaemia in early DR will cause vascular abnormalities.^16^ Thounaojam et  al reported that STZ‐rats treated with MR‐409, a growth hormone‐releasing hormone (GHRH) agonist that could prevent retinal morphological alteration, were able to sustain the survival of retinal ganglion cells. On the other hand, GHRH antagonist treatment has been shown to result in a significant alteration of the outer retinal layer and worsened retinal morphology.^17^ Therefore, preserving cell survival may prevent NPDR progression. In this study, we report that cell apoptosis was decreased after the knockdown of *Egr1*, which suggests that the down‐regulation of *Egr1* may be an effective method to sustain HRVECs viability. Moreover, diabetic patients are afflicted by a chain of vascular disorders. Early growth response protein 1 has been viewed as a key coordinator to mediate vascular dysfunction.^18^ Our results reveal that the down‐regulation of *Egr1* under high‐glucose condition decreases migration and tube formation in vitro. These results show the first experimental evidence linking *Egr1* expression status to apoptosis, migration and the formation of microvessels.

It was reported that p53 was overexpressed in diabetic patients and progressive DR, resulting in deep insights into the pathogenesis of DR.^11^ Moreover, p53 protein levels in the retinas of STZ‐induced diabetic rats were remarkably higher than those in normal rats.^2^ In addition, Kria et  al reported that p53 protein in the conjunctiva of PDR was evidently up‐regulated, while it was weak in the normal human conjunctiva.^19^ In the present study, we observed that the p53 signalling pathway is activated in DR specimens. Additionally, we show that p53 mRNA and protein levels are also up‐regulated under high‐glucose conditions. Therefore, it is reasonable to postulate that p53 may be involved in the progression of DR.

In diabetes, many ocular structures, including the retina, the cornea, the lens and the optic nerve, are affected. The microvasculature of the retina has been found to be abnormal in diabetic patients, which suggests that inhibiting the formation of microvessels seems to be an appropriate treatment strategy for DR.^16^ Moreover, p53 was found to be overexpressed in DR and to promote angiogenesis.^19^ Ghahremani et  al showed that p53 promotes the expression of VEGF and angiogenesis under hypoxic conditions.^20^ In addition, Sundaram et  al reported that p53 could promote the formation of tumour angiogenesis by promoting the expression of miR‐194.^21^

Early growth response protein 1 was found to be a major regulator of the p53 tumour suppressor pathway in order to prevent cell senescence and control replicative senescence.^5^ What is more, Das et  al held that *Egr1* may regulate the transcription and expression of p53.^22^ It was also reported that *Egr1* could ameliorate cervical cancers by strengthening radiation therapy as well as p53 signalling pathway.^23^ However, there was no information about the regulatory relationships between *Egr1 *and p53 in the DR Here, we observed that *Egr1* showed an interaction with p53 and contributed to its transcriptional activity in HRVECs. Moreover, down‐regulation of *Egr1* expression can inhibit retinal endothelial cell apoptosis, migration and microtubule formation by targeting p53, which is widely accepted as a tumour suppressor that inhibits tumour angiogenesis and promotes cell apoptosis. Obviously, our results reveal an interesting role for p53 in DR, which suggests that p53 may perform its function largely dependent on *Egr1* in DR

In conclusion, this is the first study showing the molecular mechanism of *Egr1* and p53 in DR. In vitro and in vivo studies have found that the knockdown of *Egr1* sustains endothelial cell function under high‐glucose conditions and alleviates retinal vascular dysfunction to some extent. These findings may lead to a better understanding of the progression of DR.

## 5 CONCLUSIONS

In this study, we investigated the expression and regulatory mechanism of *Egr1* in DR and found that *Egr1* was augmented after the induction of hyperglycaemia. *Egr1* regulated retinal endothelial cell apoptosis, migration and vascularization by promoting p53 transcription.

We concluded that *Egr1* was overexpressed in the retina of DR. Down‐regulation of *Egr1* partially reduced the injurious effects of hyperglycaemia on retinal vascular function via inhibiting p53 expression.

## ETHICAL APPROVAL

Animal care and experiments complied with the ARRIVE guidelines and were in accordance with the UK Animals (Scientific Procedures) Act, 1986 and associated guidelines, EU Directive 2010/63/EU for animal experiments and approved by the Institutional Animal Care and Use Committee of State Key Laboratory of Ophthalmology, Zhongshan Ophthalmic Center, Sun Yat‐sen University.

## CONFLICT OF INTEREST

No conflict of interest exits in the submission of this manuscript.

## AUTHORS' CONTRIBUTIONS

Substantial contribution to the conception and design of the work: Haocheng Ao and Lin Lu; Analysis and interpretation of the data: Haocheng Ao and Bingqian Liu; Drafting the manuscript: Haichun Li and Bingqian Liu; Revising the work critically for important intellectual content: Haocheng Ao and Lin Lu; Final approval of the work: all authors.
